# Diagnostic Value Comparison between Multislice Spiral Computerized Tomography and Magnetic Resonance Imaging under Artificial Intelligence Algorithm in Diagnosing Occult Fractures of the Knee Joint

**DOI:** 10.1155/2022/3282409

**Published:** 2022-09-27

**Authors:** Zhenghua Shu, Jun Lei, Chaoqi Ding

**Affiliations:** Department of Microsurgery, China Coast Guard Hospital of the People's Armed Police Force, Jiaxing 314000, Zhejiang, China

## Abstract

The aim of this study was to explore the application value of multislice spiral computerized tomography (MSCT) and magnetic resonance imaging (MRI) under intelligent algorithm in the diagnosis of occult fractures of the knee joint (OFKJ). 47 patients with negative X-ray examination and suspected fracture were included for this research. According to the examination methods, the patients were divided into the MSCT group and MRI group. The diagnostic results of the two methods were compared, and then compared with the traditional algorithm to explore their superiorities. The results demonstrated that the algorithm applied in this study had a clearer segmentation than traditional algorithms, and it run significantly faster than other algorithms. The results of MSCT, MRI, and pathological examination were all different, but which was of no statistical significance, *P* > 0.05. The specificity, accuracy, sensitivity, positive predictive value (PPV), and negative predictive value (NPV) of MSCT were 83%, 96%, 94%, and 98%, respectively; and its coincidence rate, missed diagnosis rate, and misdiagnosis rate were 98.20%, 1.60%, and 0.20%, respectively. Compared with MRI, the differences were significant statistically, *P* < 0.05. The segmentation effect of MSCT was closer to the standard segmentation, with the higher efficiency. MSCT under the intelligent algorithm produced the better diagnostic performance and the higher detection rate than MRI in diagnosing OFKJ. It could be used for clinical auxiliary diagnosis and evaluation of OFKJ, deserving an application value.

## 1. Introduction

In daily life, because the knee joint is composed of cancellous bones and undertakes a large amount of activity, the articular surface of the tibial plateau is tilted backward, the surface of the femoral condyle is flexed, and the femoral condyle and the patella overlap each other. Thus, it is very easy to fracture due to violence. Occult fractures of the knee joint (OFKJ) are a type of fracture in which the trabecular phalanx is broken; it is negative in normal X-ray examination but there is the bone trauma actually [1]. The knee joint is prone to fracture under external force, and occult fractures are also pretty common in clinical practice, with the main clinical manifestations of local pain and limited motion of the knee joint [2]. Untimely treatment of such fractures can lead to cortical rupture further, resulting in bone defects, pain, and even degenerative osteoarthritis and other sequalae, which lower the quality of life of patients. Therefore, the improvement of the early diagnosis rate of occult fractures has a positive effect on improving prognosis. The diagnosis of fractures often relies on imaging examinations [3].

X-ray, as the first choice for clinical fracture examination, has the advantages of being cheap and convenient. But it is not ideal for the diagnosis of split fractures, joint avulsion fractures, and slightly displaced fractures, with a high rate of missed diagnosis [4]. Magnetic resonance imaging (MRI) has high resolution for the soft tissue and is highly sensitive to abnormal changes in cartilages and bones. It has the multiplane imaging functions of axial, sagittal, and coronal planes, that conventional computerized tomography (CT) and X-ray imaging lack, thereby reducing the missed diagnosis rate and the misdiagnosis rate [5]. MRI can also show the articular cartilage damage, bone marrow edema, joint effusion, and other complicated lesions through the sagittal, coronal, and cross-sectional upper imaging, thereby increasing the diagnosis rate of OFKJ [6]. Multislice spiral computed tomography (MSCT) has the advantages of easy operation and high accuracy for clinical diagnosis and is a common imaging method for diagnosing occult fractures currently [7]. MSCT adopts the volumetric acquisition method, which can not only scan thin layers, but also increase the scope of a single examination significantly. It has a high spatial resolution with obvious advantages in the diagnosis of trauma such as fractures [8]. In addition, MSCT has high density resolution without overlapping images. This allows the comprehensive observation and analysis of the fracture types and morphology, the degree of articular surface involvement can be determined accurately, and occult fractures can also be detected [9]. A more effective basis is offered for the evaluation of the fracture types, sclerotin morphology, and joint correspondence [10]. In addition, the MSCT three-dimensional reconstruction examination technology can improve the spatial resolution of images significantly and display the joint ligaments, tendons, meniscus, and trabecular bone structures clearly [11].

With the continuous advancement of CT hardware instruments, the theory of CT image reconstruction has also undergone a series of revolutions. In the early days, parallel beam iterative algorithms were used for reconstruction in CT systems [12]. However, due to the slow scanning speed and the limitation of computer operation speed at that time, this kind of algorithms was extremely inefficient and time-consuming for calculation and was gradually replaced by the fan-beam filter back-projection algorithm. The filtering back-projection algorithm has high computational efficiency and is easy to implement, so it is widely used in practical products and has been extended to spiral CT [13]. To the 21st century, various artificial intelligence algorithms have greatly improved the computing power of computers, among which iterative algorithms have once again drawn people's attention. Although its calculating time is still long, it is within the tolerable range and has some incomparable characteristics of other algorithms. For example, it can suppress noise effectively and perform reconstruction in the case of limited scanning angle or partial data missing. Furthermore, the precise reconstruction technology is being improved constantly, and corresponding algorithms for circular trajectories, spiral trajectories, and general trajectories have been developed [14]. Precise reconstruction technology can reconstruct three-dimensional volume data under the smallest radiation dose directly, and the image resolution is extremely high; but due to the influence of calculating time and other factors, this technology has not been put into practical products yet.

In this study, patients with suspected fractures and negative X-ray examinations were included, and the artificial intelligence algorithm was applied to reconstruct MSCT images accurately. Compared with MRI examination results, its application value was studied in diagnosing OFKJ. Data and theoretical support were provided for the diagnosis and treatment of OFKJ in the future.

## 2. Research Methods

### 2.1. Objects

Forty-seven patients with suspected fractures as well as negative result of X-ray examination, who were admitted to the hospital from June 2019 to December 2021, were selected for this research. There were 32 males and 15 females, aged 22–58 years and (43.4 ± 4.7) years on average. Their course of disease was counted as 1–5 days, with (2.6 ± 0.2) days averagely. The patients were divided into the MSCT group and MRI group with different examination methods. The patients and their families singed the written informed consent, and this study had been approved by ethics committee of the hospital. The inclusion criteria include the following: clinical manifestations included abnormal knee joint movement, swelling, and pain. No fracture sign was detected by the X-ray examination. They were confirmed with knee fracture by MSCT. The exclusion criteria include the following: patients were complicated with degenerative diseases of the knee joint, cognitive impairment, or mental illness.

### 2.2. Methods for Examination and Evaluation

The multislice spiral CT scanner was used. The tube voltage was 120 kV, the tube current was 250 mAs, the pitch was 0.8, and the slice distance/slice thickness was 4 mm. The patient was arranged to take supine position with the foot first, and the scanning area was from 5 cm above the femoral condyle to 5 cm below the tibial condyle. The data were obtained for thinning reconstruction (with slice interval of 0.5–1.0 mm, slice thickness of 0.75–1.5 mm, window value of the bone, and convolution kernel of B50–70). Then, the data were sent to the workstation for CT three-dimensional reconstruction.

MRI scanner was also applied. Routine scanning was performed, including the coronal fat-suppression T2 weighted imaging (T2WI) (time of echo (TE): 87, time of repetition (TR): 4500), and sagittal T1 weighted imaging (T1WI) (TE: 17 and TR: 450). Some parts were additionally scanned in the axial plane of proton density weighted imaging fat-suppression (PDWI-FS), T2WI, and T1WI. The layer distance was 0.5 mm, the layer thickness was 4 mm, and the number of excitations was 2.

Evaluation criteria were formulated as follows: 2 senior radiologists reviewed and analyzed the imaging signs and reached a consensus diagnosis. (1) MSCT images were accompanied by fracture line shadows or bone continuity factures, and the displaced fracture was consistent with local bone defect. (2) MRI images showed irregular linear low signal or bone cortical fractures in the cancellous area under T1WI, and the corresponding layer of T2WI showed the mixed slightly high or high signal.

Observation indicators were composed of the following: (1) The detection rate of the two diagnostic methods was compared. Detection rate = actual number of detected patients/total number of objects × 100.0%. (2) The diagnostic performance of the two methods was also compared. Specificity = true negatives/(true negatives + false positives) × 100%. Sensitivity = true positives/(true positives + false negatives) × 100%. Negative predictive value (NPV) = true negatives/(true negatives + false negatives) × 100%. Positive predictive value (PPV) = true positive/(true positive + false positive) × 100%. (3) The coincidence rate, missed diagnosis rate, and misdiagnosis rate of the two diagnostic methods were also compared. Coincidence rate = (true positives + true negatives)/(true positives + false positives + false negatives + true negatives). Missed diagnosis rate = false negative/(true negative + false positive). Misdiagnosis rate = false positive/(true negative + false positive).

### 2.3. MSCT Reconstruction Algorithm

The steps of approximate reconstruction of multisource CT mainly consisted of projection data acquisition, reconstruction of tomographic data interpolation, interpolation of data filtering, and two-dimensional fan-beam filtering back-projection reconstruction [15].

During scanning of fixed-pitch spiral CT, the bed moved in a straight line at a constant speed along the *Z*-axis, and the pitch of the spiral scanning trajectory was fixed and did not change with time [16]. The motion trajectory of the *i*-th *X* source could be described as

(1) $$\begin{array}{c} x_{i}=\rho ∙\cos\;\left(\omega t+\emptyset_{i}\right)\text{,}\\ y_{i}=\rho ∙\sin\;\left(\omega t+\emptyset_{i}\right)\text{,}\\ Z_{i}=\frac{h∙\omega t}{2\pi }\text{,} \end{array}$$

where *ρ* is the radius of the spiral line, and *ω* is the angular velocity of the X-ray source and the detector array rotating; ∅_*i*_ is the initial phase of the *i*-th X-ray source, and *h* is the bed advance distance of the X-ray source and the detector array per rotation.

Before reconstruction, the reconstruction faultage position *Z*_*R*_ was firstly determined. The angle *β*_*R*_ that the *X* source rotated from the starting position to the reconstruction position was calculated through *β*_*R*_=*ωt*_*R*_=2*πZ*_*R*_/*h*.

Then, the plane fan-beam projection data necessary to reconstruct the tomographic image at *Z*_*R*_ were calculated by interpolation in the range of *β* ∈ [*β*_*R*_, *β*_*R*_+2*π*]. The basic idea of interpolation is similar to the 180MLI interpolation algorithm of single-source spiral CT; the difference lies in that the cross-spiral projection data belonging to different *X* sources are used to perform linear interpolation in the *Z*-axis direction. (*β*, *γ*, *q*) denoted each projected ray in the fan beam, and pairs (*β*, *γ*) denoted the X-rays in the fan beam. *q* was the *q*-th layer detector corresponding to the *X* source. The corresponding X-rays (*β*′, *γ*′, *q*′) parallel to (*β*, *γ*, *q*) in all *X* sources satisfied equation (2) approximately (where *k* is an integer).

(2) $$\begin{array}{c} \left\{\begin{array}{c} \beta^{\prime }=\beta +2k\pi -\frac{\pi i}{N}\\ \gamma^{\prime }=\gamma \end{array}\right.\;or\;\left\{\begin{array}{c} \beta^{\prime }=\beta +2\gamma +\left(2k-1-\frac{i}{N}\right)\pi \\ \gamma^{\prime }=-\gamma \end{array}\right.,i=1∼N,q^{\prime }=1-Q\text{,} \end{array}$$

*Z*_*i*_(*β*′, *q*′) was set to represent the *Z*-axis position of the i-th *X* source corresponding to the *q′*-layer detector under the angle parameter *β′*. Then, the equations below are defined as

(3) $$\begin{array}{c} Z_{A}=Z\left|\left(Z_{i}\left(\beta^{\prime },q^{\prime }\right)\geq Z_{R}\right)\cap \left(\left|Z-Z_{R}\right|=\min\;\left(\left|Z_{i}\left(\beta +2k\pi -\frac{\pi i}{N},q^{\prime }\right)-Z_{R}\left|,\right.\left|Z_{i}\left(\beta +2\gamma +\left(2k-1-\frac{i}{N}\right)\pi ,q^{\prime }\right)-Z_{R}\right|\right.\right)\right)\right.,i=1∼N,q^{\prime }=1-Q\text{,} \end{array}$$

(4) $$\begin{array}{c} Z_{B}=Z\left|\left(Z_{i}\left(\beta^{\prime },q^{\prime }\right)\leq Z_{R}\right)\cap \left(\left|Z-Z_{R}\right|=\min\;\left(\left|Z_{i}\left(\beta +2k\pi -\frac{\pi i}{N},q^{\prime }\right)-Z_{R}\left|,\right.\left|Z_{i}\left(\beta +2\gamma +\left(2k-1-\frac{i}{N}\right)\pi ,q^{\prime }\right)-Z_{R}\right|\right.\right)\right)\right.,i=1∼N,q^{\prime }=1-Q\text{,} \end{array}$$

*G*_*i*_(*β*′, *γ*′, *q*′) is also set as the projection data of the *i*-th *X* source corresponding to the parameter (*β*′, *γ*′, *q*′), then the projection data corresponding to *Z*_*A*_ and *Z*_*B*_ are expressed as equations (5) and (6), respectively.

(5) $$\begin{array}{c} G_{A}\left(\beta ,\gamma \right)=G_{i}\left(\beta^{\prime },\gamma^{\prime },q^{\prime }\right)\left|\left(Z_{i}\left(∎\right)\geq Z_{R}\right)\cap \left[\left(\left(Z_{i}\left(\beta +2k\pi -\frac{\pi i}{N},q^{\prime }\right)=Z_{A}\right)\cap \left(\gamma^{\prime }=\gamma \right)\right)\cup \left(\left(Z_{i}\left(\beta +2\gamma +\left(2k-1-\frac{i}{N}\right)\pi ,q^{\prime }\right)=Z_{A}\right)\cap \left(\gamma^{\prime }=-\gamma \right)\right)\right]\right.,i=1∼N,q^{\prime }=1-Q\text{,} \end{array}$$

(6) $$\begin{array}{c} G_{B}\left(\beta ,\gamma \right)=G_{i}\left(\beta^{\prime },\gamma^{\prime },q^{\prime }\right)\left|\left(Z_{i}\left(∎\right)\leq Z_{R}\right)\cap \left[\left(\left(Z_{i}\left(\beta +2k\pi -\frac{\pi i}{N},q^{\prime }\right)=Z_{B}\right)\cap \left(\gamma^{\prime }=\gamma \right)\right)\cup \left(\left(Z_{i}\left(\beta +2\gamma +\left(2k-1-\frac{i}{N}\right)\pi ,q^{\prime }\right)=Z_{B}\right)\cap \left(\gamma^{\prime }=-\gamma \right)\right)\right]\right.,i=1∼N,q^{\prime }=1-Q\text{.} \end{array}$$

Therefore, the value of the projection ray could be worked out by linear interpolation via equation (7) with the parameter (*β*, *γ*) at the *Z*_*R*_ faultage.

(7) $$\begin{array}{c} G\left(\beta ,\gamma \right)=w∙G_{A}\left(\beta ,\gamma \right)+\left(1-w\right)∙G_{B}\left(\beta ,\gamma \right)\text{.} \end{array}$$

*w*=(*Z*_*A*_ − *Z*_*R*_) ÷ (*Z*_*A*_ − *Z*_*B*_), and finally, the tomographic image was reconstructed using the fan-beam plane reconstruction (4). Using the multiplane reconstruction technique, the three-dimensional volume data were reconstructed with a series of tomographic images.

In more general cases, to meet special scanning needs such as real-time tracking of contrast agent clumps in CT angiography, the bed moved linearly with variable speed along the *Z* axis. The scanning trajectory thus was no longer a standard spiral line, as its pitch changed with time. Similar to equation (1), the scanning trajectory equation is defined as

(8) $$\begin{array}{c} x_{i}=\rho ∙\cos\;\left(\omega t+\emptyset_{i}\right)\text{,}\\ y_{i}=\rho ∙\sin\;\left(\omega t+\emptyset_{i}\right)\text{,}\\ y_{i}=\frac{\int_{0}^{t}h\left(\omega \tau \right)\omega \;d\tau }{2\pi }\text{,} \end{array}$$

(*β*, *γ*, *q*) still represented a projection ray in the fan beam. After the reconstruction position *Z*_*R*_ was determined, the above equations were utilized to calculate the angle *β*_*R*_=*ωt*_*R*_ used by one of the *X* sources rotating from the starting position to the reconstructed faultage. With this *X* source as a reference, subsequent interpolation, and reconstruction were then performed.

The *Z*-axis interpolation algorithm of multisource variable-pitch spiral CT needed to take the more general *Z*-axis interpolation of cross-spiral, multilayer projection data into account when the pitch varied [17]. During interpolation, 2 projection rays located on both sides of *Z* and closest to *Z*_*R*_ were sought among all projection rays parallel to ray (*β*, *γ*). The selected data could come from detectors of the same source, but also detectors corresponding to different sources. In Figure 1, the scanning trajectories of two *X* sources are shown. It was assumed that each *X* source corresponded to 4 rows of detectors, and then the two bold lines at A and B in the figure represented the selected projection data. These two rows of data were expressed by *G*_*A*_(*β*_1_, *γ*_1_, *q*_1_) and *G*_*B*_(*β*_2_, *γ*_2_, *q*_2_), respectively.

Equation (2) was taken as the approximate judgment condition for ray parallel, *G*_*i*_(*β*, *γ*, *q*) represented the projection data corresponding to the *i*-th *X* source. *z*_*i*_(*β*, *q*) indicated the corresponding *Z*-axis position of the *q*-th layer detector after the *i*-th *X* source rotating through *β*. The 4 sets are defined as equations (9)–(12).

(9) $$\begin{array}{c} G_{2\pi }^{-}\left(\beta_{2\pi }^{-},\gamma_{2\pi }^{-},q_{2\pi }^{-}\right)=G_{i}\left(\beta^{\prime },\gamma^{\prime },q\right)\left|\min\;\left(Z_{R}-z_{i}\left(\beta_{i}^{\prime },q\right)\right)\right.{,Z}_{R}\geq z_{i}\left(\beta_{i}^{\prime },q\right)\\ \gamma^{\prime }=\gamma ,\beta^{\prime }=\beta +2k\pi -\frac{j\pi }{N},j\in \left\{1,\ldots ,N\right\}\text{,} \end{array}$$

(10) $$\begin{array}{c} G_{\pi }^{-}\left(\beta_{\pi }^{-},\gamma_{\pi }^{-},q_{\pi }^{-}\right)=G_{i}\left(\beta^{\prime },\gamma^{\prime },q\right)\left|\min\;\left(Z_{R}-z_{i}\left(\beta_{i}^{\prime },q\right)\right)\right.,Z_{R}\geq z_{i}\left(\beta_{i}^{\prime },q\right)\\ \gamma^{\prime }=-\gamma ,\beta^{\prime }=\beta +2k\pi -\pi -\frac{j\pi }{N},j\in \left\{1,\ldots ,N\right\}\text{,}\\ \gamma^{\prime }=\gamma ,\beta^{\prime }=\beta +2k\pi -\frac{j\pi }{N},j\in \left\{1,\ldots ,N\right\}\text{,}\\ \gamma^{\prime }=-\gamma ,\beta^{\prime }=\beta +2k\pi -\pi -\frac{j\pi }{N},j\in \left\{1,\ldots ,N\right\}\text{.} \end{array}$$

(11) $$\begin{array}{c} G_{2\pi }^{+}\left(\beta_{2\pi }^{+},\gamma_{2\pi }^{+},q_{2\pi }^{+}\right)=G_{i}\left(\beta^{\prime },\gamma^{\prime },q\right)\left|\min\;\left(z_{i}\left(\beta_{i}^{\prime },q\right)-Z_{R}\right)\right.,Z_{R}\leq z_{i}\left(\beta_{i}^{\prime },q\right)\\ \gamma^{\prime }=\gamma ,\beta^{\prime }=\beta +2k\pi -\frac{j\pi }{N},j\in \left\{1,\ldots ,N\right\}\text{,}\\ \gamma^{\prime }=-\gamma ,\beta^{\prime }=\beta +2k\pi -\pi -\frac{j\pi }{N},j\in \left\{1,\ldots ,N\right\}\text{.} \end{array}$$

(12) $$\begin{array}{c} G_{\pi }^{+}\left(\beta_{\pi }^{+},\gamma_{\pi }^{+},q_{\pi }^{+}\right)=G_{i}\left(\beta^{\prime },\gamma^{\prime },q\right)\left|\min\;\left(z_{i}\left(\beta_{i}^{\prime },q\right)-Z_{R}\right)\right.,Z_{R}\leq z_{i}\left(\beta_{i}^{\prime },q\right)\\ \gamma^{\prime }=-\gamma ,\beta^{\prime }=\beta +2k\pi -\pi -\frac{j\pi }{N},j\in \left\{1,\ldots ,N\right\}\text{.} \end{array}$$

From the above four sets, *G*_*A*_(*β*_1_, *γ*_1_, *q*_1_) and *G*_*B*_(*β*_2_, *γ*_2_, *q*_2_) were calculated as equations (13) and (14).

(13) $$\begin{array}{c} G_{A}\left(\beta_{1},\gamma_{1},q_{1}\right)=\left\{\begin{array}{c} G_{2\pi }^{-}\left(\beta_{2\pi }^{-},\gamma_{2\pi }^{-},q_{2\pi }^{-}\right),Z_{R}-z\left(\beta_{2\pi }^{-},q_{2\pi }^{-}\right)\leq Z_{R}-z\left(\beta_{\pi }^{-},q_{\pi }^{-}\right)\\ G_{\pi }^{-}\left(\beta_{\pi }^{-},\gamma_{\pi }^{-},q_{\pi }^{-}\right),else \end{array}\right)\text{,} \end{array}$$

(14) $$\begin{array}{c} G_{B}\left(\beta_{2},\gamma_{2},q_{2}\right)=\left\{\begin{array}{c} G_{2\pi }^{+}\left(\beta_{2\pi }^{+},\gamma_{2\pi }^{+},q_{2\pi }^{+}\right),z\left(\beta_{2\pi }^{+},q_{2\pi }^{+}\right)-Z_{R}\leq z\left(\beta_{\pi }^{+},q_{\pi }^{+}\right){-Z}_{R}\\ G_{\pi }^{+}\left(\beta_{\pi }^{+},\gamma_{\pi }^{+},q_{\pi }^{+}\right),else \end{array}\right)\text{.} \end{array}$$

The projected data G(*β*, *γ*) after interpolation was further calculated through

(15) $$\begin{array}{c} G\left(\beta ,\gamma \right)=w∙G_{A}\left(\beta_{1},\gamma_{1},q_{1}\right)+G_{B}\left(\beta_{2},\gamma_{2},q_{2}\right)-w∙G_{B}\left(\beta_{2},\gamma_{2},q_{2}\right)\text{.} \end{array}$$

In equation (15), *w*=*z*(*β*_2_, *q*_2_) − *Z*_*R*_/*z*(*β*_2_, *q*_2_) − *z*(*β*_1_, *q*_1_). After *β* took all the projection angles in (*β*_*R*_, *β*_*R*_+2*π*), all the projection data necessary to reconstruct the tomographic image at *Z*_*R*_ could be obtained.

### 2.4. Image Reconstruction Evaluation

For Dice similarity coefficient, *M* was set as the set of image pixels that were the gold standard for manual segmentation, and *N* was the set of all image pixels obtained by the semiautomatic or automatic segmentation algorithm. Then, the Dice similarity coefficient could be expressed as

(16) $$\begin{array}{c} Dice\left(M,N\right)=\frac{2\left|M∁N\right|}{\left|M\right|+\left|N\right|}\text{.} \end{array}$$

If *M* and *N* did not intersect, the Dice similarity coefficient was 0; if *M* and *N* were completely intersected, the Dice similarity coefficient was 1.

The efficiency in this study referred to the time spent by the computer in the calculation and execution because the time consumed by each sample was difficult to count in the research process and there were errors for each operation.

### 2.5. Statistical Methods

SPSS 22.0 was applied for data analysis. The enumeration data were expressed as a rate, and the pairwise comparisons were performed using the *χ*^2^ test. A difference was considered as statistically significant at *P* < 0.05.

## 3. Research Results

### 3.1. Image Reconstruction Results

The segmentation of bone tissue sections of the knee joint is displayed in Figure 2.  Figure 2(a) was the original image, while Figure 2(b) was the reconstructed image. It could be observed from Figure 2 that when the foreground was complex and scattered, the number of seed points that needed to be marked by the traditional algorithm increased obviously with more interferences. The algorithm in this study had a clear segmentation and the better effect. Meanwhile, the algorithm here is more efficient in image segmentation, which is shown as Figure 3.

From equation (16), the greater the Dice similarity coefficient, the smaller the difference between the image segmentation result and the standard segmentation result. When the Dice similarity coefficient was smaller, the difference between the two was larger. Therefore, as represented in Figure 4, the algorithm applied had a great improvement in the effect of image segmentation compared with the traditional algorithm.

### 3.2. Comparison of the Diagnosis of OFKJ by Two Examination Methods

Postoperative pathological examination confirmed that, among the 47 patients, there were 7 cases with medial femoral condyle fractures, 11 cases with lateral femoral condyle fractures, 10 cases with medial tibial condyle fractures, 8 cases with lateral tibial condyle fractures, 9 cases with central tibial plateau fractures, 6 cases with tibial condylar spine fractures, 7 cases with patella fracture, and 7 cases with fibular head factures. The preoperative MSCT showed that there were 6, 8, and 6 cases with medial femoral condyle fracture, tibial medial condyle fracture, and patella fracture, respectively. Compared with the results of pathological examination, a difference was found but of no statistical significance, *P* > 0.05. MRI examination showed that, medial condyle fractures, lateral femoral condyle fractures, medial tibial condyle fractures, central tibial plateau fractures, patellar fractures, and fibular head fractures occurred in 3, 8, 6, 6, 4, and 5 cases, respectively. Similarly, the difference compared with pathological examination results was not significant statistically, *P* > 0.05 (Figure 5).

### 3.3. Comparison of the Diagnostic Performance for OFKJ between the Two Examination Methods

The specificity, sensitivity, PPV, and NPV of MSCT were 83%, 96%, 94%, and 98%, respectively, for the diagnosis of OFKJ; the specificity, sensitivity, PPV, and NPV of MRI were 66%, 82%, 46%, and 83%, respectively. As the two examination methods were compared, the differences in the diagnostic performance were significant statistically, *P* < 0.05 (Figure 6).

### 3.4. Comparison of the Detection Rate for OFKJ between the Two Examination Methods

The coincidence rate, missed diagnosis rate, and misdiagnosis rate of MSCT in the diagnosis of OFKJ were 98.20%, 1.60%, and 0.20%, respectively; those of MRI were 86.80%, 8%, and 5.20%, respectively. In the comparison of the two methods, the differences in the indicators were thought to be significant statistically, *P* < 0.05 (Figure 7).

## 4. Discussion

Nowadays, MSCT technology has been widely applied in clinical practice and will still receive extensive attention for a long time in the future. With the continuous improvement of quasi-precise and precise reconstruction algorithms and the development of hardware devices, some theories at this stage may enter people's lives soon. The introduction of precise reconstruction techniques can bring image quality to a higher level, with higher image resolution and fewer reconstruction artifacts [18]. The results of this study suggested that, compared with the traditional algorithms, the number of seed points needed to be marked increased remarkably in the traditional algorithms with more complex and scattered foreground, which brought more interference to the segmentation. While the algorithm in this study had the clear segmentation and the better effect. In the comparison with the segmentation under traditional algorithms, the image segmentation effect was greatly improved to be closer to the standard segmentation.

A study by Xin and Lei [19] showed that MRI and MSCT had unique advantages in the diagnosis of spinal injuries, and patients with negative X-ray results could be examined by MRI and MSCT to observe their spinal injuries. In this research, 47 patients were eventually selected with negative X-ray examination result as well as the suspected fractures. The patients were examined by the intelligent algorithm-based MSCT and MRI. In MSCT examination, 6 cases were detected with medial femoral condyle fractures, 8 cases went with tibial medial condyle fractures, and 6 cases had patella fractures. Those were different from the results of pathological examination; however, there was no statistical significance, *P* > 0.05. MRI showed that 3 cases, 8 cases, 6 cases, 6 cases, 4 cases, and 5 cases got medial femoral condyle fractures, lateral femoral condyle fractures, medial tibial condyle fractures, central tibial plateau fractures, patella fracture, and fibular head fractures, respectively. The difference compared to the pathological examination results was not of statistical significance, *P* > 0.05. The accuracy of the intelligent algorithm-based MSCT was higher; but perhaps the sample size was small, so that there was not a significant difference in the diagnosis between the two examination methods. Rolvien et al. [20] revealed that, in the diagnosis of small foreign bodies in the hands, MSCT showed a higher detection rate while MRI did not provide diagnostic benefit, similar to the findings in this study.

Relevant studies have suggested that MSCT allows to observe the correlation among adjacent structures of the knee joint in details and the fractures in various parts. Not only can the range of a single examination be improved, but thin-slice scanning can be performed efficiently. Images of various sizes at any angle and at any layer can be obtained using volume data, which are convenient for multidirectional observation and identification of damaged parts and fine cracks. It is particularly suitable for joint fractures with complex anatomical structures such as the knee joint [21]. The results of this study showed that for MSCT in the diagnosis of OFKJ, the specificity was 83%, the sensitivity was 96%, the PPV was 94%, and the NPV was 98%. The diagnostic specificity, sensitivity, PPV, and NPV were 66%, 82%, 46%, and 83%, respectively, of MRI. As the two examination methods were compared, the differences in these four indicators were significant statistically for *P* < 0.05. The coincidence rate, missed diagnosis rate, and misdiagnosis rate of MSCT in diagnosing OFKJ were 98.20%, 1.60%, and 0.20%, respectively, and were 86.80%, 8%, and 5.20%, respectively, of MRI. In comparison between the two examination methods, the differences were of statistical significance, *P* < 0.05. These were consistent with the findings of previous research studies. A diagnosis of condylar cystoid lesions of the temporomandibular joint showed that the detection rate was 100% of MSCT and 80.1% of MRI. This is consistent with the results of this research [22].

## 5. Conclusion

The results proved that, compared with the traditional algorithm, the reconstruction algorithm used in this study had a better segmentation effect, runs faster, and was more efficient. Compared with MRI in diagnosing OFKJ, the intelligent algorithm-based MSCT had the better diagnostic performance and higher detection rate. However, due to limited conditions, this research included a small sample size, and the results of some comparisons were not significantly different. Therefore, its accuracy needed to be further confirmed later. In short, MSCT under the intelligent algorithm had better detection effect in the diagnosis of OFKJ, having the application value and promotion value.

## Figures and Tables

**Figure 1:** Schematic diagram of interpolation projection.

**Figure 2:** Comparison of CT images after algorithm reconstruction. (a) Original image; (b) reconstructed image.

**Figure 3:** The running time of algorithms. Compared with traditional algorithm, ^*∗*^*P* < 0.05.

**Figure 4:** Comparison of dice values among the algorithms. ^*∗*^Compared with canny operator algorithm *P* < 0.05; #compared with simple linear iterative cluster (SLIC) algorithm, *P* < 0.05.

**Figure 5:** Comparison of diagnostic results by different methods.

**Figure 6:** Comparison of diagnostic performance between the different methods. ^*∗*^Compared with MSCT, *P* < 0.05.

**Figure 7:** Comparison of detection rates under different methods. ^*∗*^Compared with MSCT, *P* < 0.05.

## Data Availability

The data used to support the findings of this study are available from the corresponding author upon request.
